# Effect of Operating Room Nursing Management on Nosocomial Infection in Orthopedic Surgery: A Meta-Analysis

**DOI:** 10.1155/2022/4193932

**Published:** 2022-02-26

**Authors:** Yuying He, Jun Chen, Yufeng Chen, Huangjing Qian

**Affiliations:** ^1^Department of Operation Room, Taizhou Hospital of Zhejiang Province Affiliated to Wenzhou Medical University, Enze Hospital, Taizhou Enze Medical Center (Group), Taizhou 318050, Zhejiang, China; ^2^Department of Operation Room, The First Affiliated Hospital of Wenzhou Medical University, Wenzhou 325025, Zhejiang, China

## Abstract

**Objective:**

This study aimed to provide scientific management methods to prevent nosocomial infection based on the systematical evaluation of the effect of operating room nursing management on nosocomial infection in orthopedic surgery.

**Methods:**

PubMed, Web of Science, Embase, China National Knowledge Internet, and Wanfang Databases were systematically searched for relevant studies published from 2013 to 2020. In this meta-analysis, comprehensive estimates of effect size estimates and 95% confidence intervals (CIs) for nursing satisfaction and incidence of infection were obtained.

**Results:**

Twenty studies with 2962 orthopedic patients were included in the meta-analysis. The experimental group received operating room nursing management while the routine nursing management was given for the control group. Meta-results showed that, in comparison with the control group, the nursing satisfaction in the experimental group was increased (OR = 6.22, 95% CI: 4.63–8.35, *P* < 0.001), while the incidence of infection was reduced (OR = 0.20, 95% CI: 0.15–0.28, *P* < 0.001), and the differences had statistical significance.

**Conclusions:**

Operating room nursing management could reduce the incidence of infection while prevent nosocomial infection in orthopedic surgery, which could be utilized to guide the hospital management.

## 1. Introduction

In recent years, nosocomial infections have increasingly become one of the major problems faced by hospital management. Nosocomial infections are defined as infections in hospitalized patients that occur during hospitalization and after discharge, excluding infections that are already in the incubation period before or at admission [1, 2]. Nosocomial infections are already a life-threatening health problem, resulting in reduced surgery efficacy, prolonged recover time, and increased medical economic burden. Therefore, these infections have been paid more and more attention, especially in orthopedic surgery where infection is one of the most common complications and the risk of nosocomial infection is high.

Zhang et al. [3] investigated 9126 inpatients in Henan Provincial Orthopedic Hospital from 2009 to 2019 and found an average infection rate of 1.96% (176/8975). Qi et al. [4] monitored 4022 patients who underwent surgery for fracture from 2009 to 2011 and found a nosocomial infection rate of 0.94% (38/4022). These infections probably occur as a result of the orthopedic surgery with a long operation time and large wound surface, and implantation of allogeneic materials such as allogeneic bone, bone cement, steel plate, screw, and artificial joint. Additionally, patients have long postoperative recovery time staying in bed, and during this period, due to the poor blood supply to bone tissue, the condition is more serious and difficult to control once a surgical wound infection occurs [5]. Among the common microorganisms in arthroplasty infections are *coagulase-negative staphylococci*, *Staphylococcus aureus*, *aerobic Gram-negative bacilli*, etc. These microorganisms may lead to urinary tract infections, infected leg ulcers, and other hazards [6]. Therefore, it is necessary to prevent nosocomial infection in orthopedic surgery.

Drugs are often used in clinical practice to prevent and treat perioperative infections [7]. Some studies have found that proper operating room care is beneficial in reducing surgical site infections [8]. Relevant studies have shown that operating room nursing management can effectively reduce the incidence of nosocomial infection and improve nursing satisfaction, thus achieving a significant effect in preventing nosocomial infection [9]. However, current studies lack systematic evaluation of their clinical effects. Therefore, in this study, a systematic evaluation method was used to explore the prevention of nosocomial infection in orthopedic surgery by operating room nursing management, so as to achieve the effects mentioned above and to guide the hospital management.

## 2. Materials and Methods

### 2.1. Literature Retrieval

Two reviewers independently searched PubMed, Web of Science, Embase, China National Knowledge Internet (CNKI), and Wanfang databases for relevant articles related to operating room nursing management and nosocomial infections in orthopedic surgery between 2013 and 2020, without limitations of publication date and language. The following keywords were included: (“operating room nursing management” or “nursing management of operating room”), (“orthopedic surgery” or “orthopedics operation”), (“hospital infection” or “nosocomial infection”), and (“intervention effect” or “intervention outcome”).

### 2.2. Inclusion and Exclusion Criteria

Inclusion criteria: (1) study type: randomized controlled trials on the intervention effect of operating room nursing management on nosocomial infection in orthopedic surgery. (2) Study subjects: orthopedic surgery patients. (3) Intervention measures: in the experimental group, operating room nursing management was performed with the following specific measures: ① preoperative management: preoperative comprehensive evaluation for all patients and active control of their underlying diseases to prepare for surgery, restriction of movement of personnel in the operating room, and preoperative disinfection of surgical instruments. ② Nursing during surgery: closed the operating room to avoid contamination, kept the patients in a comfortable state and provided surgical guarantee, strictly controlled the number of learning personnel, maintained sufficient distance from other surgical personnel, ensured the sterility of the surgical area, and strengthened the professional quality of nursing staff to avoid the infection caused by nursing operation errors during the operation. ③ Postoperative nursing: closely monitored the vital signs of the patients, protected their surgical incision during moving them, regularly checked the incision, timely replaced the drugs, and immediately checked if infection occurred. In contrast, the control group was received routine nursing management, mainly nursing intervention given according to the actual needs of the patients and the doctor's advice. (4) Outcome outcomes: at least any one of nursing satisfaction and incidence of adverse reactions.

Exclusion criteria: (1) literature whose data could not be extracted; (2) literature that could not obtain the original text cannot be obtained; (3) literature with poor quality and missing data, and duplicate literature; (4) case report, systematic review, and animal experiment.

### 2.3. Data Extraction and Quality Evaluation

Two investigators independently reviewed and extracted information from the eligible studies, and all disagreements were resolved through discussion with a third investigator. Data extraction included basic information in the literature, type of the study method, sample size, and outcome measures. Eligible studies were evaluated for quality according to the Newcastle Ottawa Scale (NOS) [10].

### 2.4. Statistical Analysis

All data were statistically analyzed with Stata16.0 software. *Q* test and I^2^ test were utilized for evaluating heterogeneity. In case of heterogeneity (*I*^2^ < 50% and *P* > 0.05), the fixed-effects model was used; otherwise (*I*^2^ > 50% and *P* < 0.05), the random-effects model was adopted. Nursing satisfaction and incidence of adverse reactions were quantitatively expressed as odds ratio (*OR*), 95% confidence interval (CI), and *P* value. Publication bias was assessed using Egger's and Begg's tests, as well as funnel plots. Sensitivity analysis was performed to evaluate the stability of the meta-analysis results.

## 3. Results

### 3.1. Screening Results and Basic Characteristics of Included Studies

Initially, 479 articles were retrieved and then 422 were excluded based on the screening criteria. Full texts of the remaining 57 articles were read to exclude case reports, systematic reviews, and animal experiments. Finally, 20 articles were included in this meta-analysis. The screening process is shown in Figure 1. The included studies were all randomized controlled trials, with a total of 2962 subjects: 1484 in the experimental group and 1478 in the control group. The age of the patients in the experimental group was 35.8–57.7 years, while 36.1–58.5 years in the control group. The gender ratio of the experimental group (805/679) was similar to that of the control group (800/678). All studies mentioned nursing satisfaction and incidence of adverse reactions. The characteristics of the included articles are detailed in Table 1. The NOS scores of 6∼9 indicated the high methodological quality of the included studies.

### 3.2. Meta-Analysis Results

#### 3.2.1. Nursing Satisfaction

20 studies compared the nursing satisfaction between the two groups. No marked heterogeneity was found among these studies (*P*=0.883, *I*^2^ = 0.00%), so the fixed-effects model was used to combine the effect sizes. The results revealed that the postoperative satisfaction of patients in the experimental group was significantly higher than that of the control group (OR = 6.22, 95% CI: 4.63–8.35, *P* < 0.001) (Figure 2(a)).

#### 3.2.2. Incidence of Infection

All 20 studies reported the incidence of infection after postoperative care in both groups. There was no significant heterogeneity among the included studies (*P*=0.931, *I*^2^ = 0.00%), and meta-analysis was performed by the fixed-effects model. The results are shown in Figure 2(b), where the incidence rate of infection in the experimental group was significantly lower than that in the control group (OR = 0.20, 95% CI: 0.15–0.28, *P* < 0.001).

### 3.3. Publication Bias

Begg's test (*Z* = 1.85, *P*=0.064) and Egger's test (*t* = 3.86, *P*=0.001) showed no significant publication bias in nursing satisfaction between the two groups. Similarly, Begg's test (*Z* = 1.14, *P*=0.256) and Egger's test (*t* = −2.25, *P*=0.037) of incidence of infection also identified no publication bias. Furthermore, as shown in both the funnel plots of nursing satisfaction (Figure 3(a)) and infection incidence (Figure 3(b)) in orthopedic surgery patients, the included studies scattered either side of the symmetry axis in a symmetrical manner, suggesting little possibility of publication bias in this study.

### 3.4. Sensitivity Analysis

The included studies were removed one by one, and the statistical model was changed for sensitivity analysis. The results showed that the pooled effect size of nursing satisfaction did not change (OR = 6.22, 95% CI: 4.63, 8.35, *P* < 0.001), nor did the infection incidence (OR = 0.20, 95% CI: 0.15, 0.28, *P* < 0.001), suggesting that the meta-analysis had good stability. Furthermore, as shown in the sensitivity analysis plots of nursing satisfaction (Figure 4(a)) and infection incidence (Figure 4(b)), the effect size of each study fluctuated above and below the estimate, indicating that this meta-analysis had high reliability.

## 4. Discussion

Operating room nursing management is a crucial link in the whole process of surgery, which significantly affects postoperative rehabilitation. To reduce the nosocomial infection rate of surgical patients has become the focus on hospital management, especially orthopedic surgery. The operation time of orthopedic surgery is generally longer than two hours, accompanied by large surgical wounds, more invasive procedures and hemorrhage, and requiring long rehabilitation time. Due to the above factors, the nosocomial infection rate of orthopedic surgery is high [31]. Nosocomial infection will deteriorate the condition, thus prolonging hospital stays and increasing the economic, physical, and psychological burden on patients. Therefore, an in-depth study of interventions for nosocomial infections is necessary, especially in orthopedic surgery.

The intervention measures adopted in this paper include preoperative management, nursing during surgery, and postoperative nursing. First, preoperative management referred to preoperative comprehensive evaluation for all patients and active control of their underlying diseases to prepare for surgery, restriction of movement of personnel in the operating room, and preoperative disinfection of surgical instruments. Second, during surgery, we closed the operating room to avoid contamination, kept the patients in a comfortable state and provided surgical guarantee, strictly controlled the number of learning personnel, maintained sufficient distance from other surgical personnel, ensured the sterility of the surgical area, and strengthened the professional quality of nursing staff to avoid the infection caused by nursing operation errors during the operation. Third, after surgery, we closely monitored the vital signs of the patients, protected their surgical incision during moving them, regularly checked the incision, timely replaced the drugs, and immediately checked if infection occurred. All 20 studies reported the nursing satisfaction and the incidence rate of infection in the two groups. These outcome measures were extracted and comprehensive analyzed. The results showed that, in comparison with the control group, the nursing satisfaction in the experimental group was increased while the incidence of infection was reduced.

Other relevant studies have further proposed specific principles and models of operating room nursing. Chunhua et al. [32] proposed the application of 10S management in operating room nursing, including ten principles: sort (SEIRI), set in order (SEITON), sustain (SHITSUKE), standardize (SEIKETSU), sweeping (SEIS0), saving (SAVING), safety (SAFETY), habit (Shiukanka) adherence (Shikoku), and speed (SPEED). Fu et al. [33] demonstrated that the implementation of failure mode and effect analysis during surgery could effectively standardize the process of medical staff, thus improving the quality of operating room nursing, ensuring medical safety, and gaining recognition of patents more likely. Waiwaiet al. [34] believed that the application of a PDCA cycle management method in operating room nursing management had a significant effect in reducing the incidence of adverse reactions, improving patient satisfaction and comprehensive score of the operating room, which was worth popularizing and applying in operating room management. However, there are more issues to consider in clinical practice such as the input and effectiveness of nursing management. That is, the nursing management system needs to be developed in the context of the actual situation.

This meta-analysis still has the following limitations: first, the included studies are all Chinese literature, and the study location was also in China. Studies from other countries were not included, potentially leading to a language bias. Second, the search time of this paper was short, and only 20 articles were included. The sample size was relatively small and the results might be biased. Third, most of the literature has not mentioned the grouping method and could not determine whether its method was randomized. At last, there was no blind method in the included studies, and it was difficult to set blind because the intervention measure of the study was surgery. Different surgical options in the included studies may affect the outcome measures.

## 5. Conclusion

In summary, operating room nursing management, including preoperative management, nursing during surgery, and after surgery, can effectively reduce the infection incidence and increase the patient's nursing satisfaction.

## Figures and Tables

**Figure 1:** Flow chart of study selection.

**Figure 2:** Forest plots of nursing satisfaction (a) and incidence of infection (b) in two groups of orthopedic surgery patients.

**Figure 3:** Funnel plots of nursing satisfaction (a) and incidence of infection (b) in two groups of orthopedic surgery patients.

**Figure 4:** Sensitivity analysis of nursing satisfaction (a) and incidence of infection (b) in two groups of orthopedic surgery patients.

**Table 1:** Basic characteristics of inclusion in the literature.

Study	Year	Sample time (year.month)	Cases treat/Con	Age (years)		Sex (male/female)		Study design	NOS score	Outcome measures
				Treat group	Con group	Treat group	Con group			
Hongyan [11]	2019	2018.2∼2019.2	50/50	41.2 ± 1.1	44.1 ± 2.2	21/29	20/30	RCT	6	① + ②
Jinxiang [12]	2019	2017.1∼2018.6	60/60	46.8 ± 4.9	47.2 ± 5.4	33/27	36/24	RCT	6	① + ②
Lei [13]	2019	2016.3∼2018.11	39/39	51.27 ± 2.38	51.242 ± 2.35	19/20	18/21	RCT	7	① + ②
Du [14]	2020	2017.5∼2018.5	150/150	57.7 ± 4.6	58.5 ± 5.7	82/68	73/77	RCT	8	① + ②
Jun [15]	2019	2017.5∼2018.5	60/60	35.9 ± 6.9	35.3 ± 7.3	38/22	39/21	RCT	7	① + ②
Jing [16]	2019	2017.1∼2018.12	43/43	40.5 ± 22.5	41.0 ± 23.0	27/16	26/17	RCT	6	① + ②
Zhang Minhua [17]	2018	2017.1∼2017.8	32/32	35.8 ± 5.2	36.1 ± 4.1	17/15	20/12	RCT	6	① + ②
Tianxiao [18]	2017	2015.10∼2017.4	63/63	54.66 ± 2.37	53.27 ± 2.54	33/30	31/32	RCT	7	① + ②
Chao [19]	2020	2018.1∼2019.10	80/80	44.02 ± 1.57	43.98 ± 1.55	46/34	47/33	RCT	6	① + ②
Xiaowei [20]	2020	2018.10∼2019.11	30/30	50.2 ± 2.1	45.5 ± 2.5	17/13	16/14	RCT	8	① + ②
Ruiling [21]	2018	2017.1∼2018.1	43/42	49.8 ± 2.1	48.7 ± 1.9	20/23	23/19	RCT	7	① + ②
Hui and Lixia [22]	2019	2016.1∼2018.1	100/100	44.5 ± 2.8	44.8 ± 2.3	57/43	59/41	RCT	6	① + ②
Wen [23]	2017	2014.2∼2017.2	50/50	53.23 ± 4.21	53.11 ± 4.08	29/21	28/22	RCT	7	① + ②
Sha [24]	2020	2018.9∼2019.7	61/60	44.5 ± 23.5	45 ± 22	30/31	32/28	RCT	7	① + ②
Yanling [25]	2016	2015.4∼2016.3	157/153	41.3 ± 7.1	40.9 ± 7.4	90/67	84/69	RCT	7	① + ②
Ying [26]	2019	2017.12∼2018.11	44/44	43.12 ± 4.30	42.37 ± 4.22	25/19	24/20	RCT	6	① + ②
Ta et al. [27]	2018	2016.6∼2018.1	72/72	42.87 ± 3.24	42.39 ± 3.11	40/32	41/31	RCT	7	① + ②
Zhanggui [28]	2020	2016.6∼2018.1	71/71	42.87 ± 3.24	42.39 ± 3.11	40/31	40/31	RCT	9	① + ②
Bingbing and Lingzhi [29]	2017	2015.3∼2016.3	219/219	49.4 ± 4.8	49.1 ± 5.1	110/109	111/108	RCT	8	① + ②
Yingying [30]	2016	2014.1∼2016.1	60/60	38.7 ± 2.1	38.1 ± 2.5	31/29	32/28	RCT	7	① + ②

Note. Treat: treatment; Con: control; RCT: randomized controlled trial; NR: not reported; ①: nursing satisfaction of patients; ②: incidence of infection.

## Data Availability

The data used to support the findings of this study are available from the corresponding author upon request.
